# A lightweight ground crack rapid detection method based on semantic enhancement

**DOI:** 10.1016/j.heliyon.2024.e34782

**Published:** 2024-07-17

**Authors:** Bing Yi, Qing Long, Haiqiao Liu, Zichao Gong, Jun Yu

**Affiliations:** a School of Materials and Chemical Engineering, Hunan Institute of Engineering, 411104, Hunan, China; b School of Electrical and Information Engineering, Hunan Institute of Engineering, 411104, Hunan, China; c Graduate School of Hunan University of Engineering, 411104, Hunan, China

**Keywords:** Deep learning, Crack detection, Pavement maintenance, Semantic enhancement

## Abstract

To address the issue of detecting complex-shaped cracks that rely on manual, which may result in high costs and low efficiency, this paper proposed a lightweight ground crack rapid detection method based on semantic enhancement. Firstly, the introduction of the Context Guided Block module enhanced the YOLOv8 backbone network, improving its feature extraction capability. Next, the incorporation of GSConv and VoV-GSCSP was introduced to construct a lightweight yet efficient neck network, facilitating the effective fusion of information from multiple feature maps. Finally, the detection head achieved more precise target localization by optimizing the probability around the labels. The proposed method was validated through experiments on the public dataset RDD-2022. The experimental results demonstrate that our method effectively detects cracks. Compared to YOLOv8, the model parameters have been reduced by 73.5 %, while accuracy, F1 score, and FPS have improved by 6.6 %, 4.3 %, and 116, respectively. Therefore, our proposed method is more lightweight and holds significant application value.

## 1 Introduction

In chemical production and transportation environments, large oil tankers play a crucial role in transportation tasks, where road safety is paramount to ensure their smooth operation. However, road surface cracks pose a serious threat to tanker safety. Accidents caused by road surface cracks can lead to major safety incidents and environmental pollution. Moreover, poor road conditions bring various safety hazards and result in additional economic losses. According to the National Highway Traffic Safety Administration (NHTSA) data, approximately 16 % of traffic accidents are caused by road conditions [1]. Timely detection of road damage is essential to maintain traffic safety and provide basis for subsequent road repairs and maintenance. Most detection models require significant computational resources and storage space, making them impractical for inference on resource-constrained devices. Lightweight models can reduce model size and computational complexity, thereby improving running speed and performance [2]. Therefore, lightweight road damage detection technology can significantly enhance detection efficiency and reduce labor costs, while also playing a crucial role in ensuring driving safety and extending road lifespan.

In recent years, with the development of deep learning, methods for crack detection based on deep learning have become a trend. These methods can automatically extract various features of cracks. Based on deep learning, crack detection methods can be divided into semantic segmentation methods and object detection methods [3]. König et al. [4] addressed surface crack segmentation challenges by focusing on the decoder part of semantic segmentation, introducing different encoder strategies and data augmentation techniques. He et al. [5] proposed an unmanned aerial vehicle (UAV) road crack detection algorithm using MUENet, incorporating Main and Auxiliary Dual Path Modules (MADPM), Uneven Fusion Structure (TI-UFS), and E-SimOTA strategy to achieve efficient and precise detection and differentiation of cracks. However, this method is limited to specific geographical areas or environments, with restricted generalization capability of its results. Djenouri et al. [6] introduced an intelligent system based on graph convolutional neural networks, utilizing Scale-Invariant Feature Transform (SIFT) for image feature extraction and generating graphs by analyzing correlations between SIFT features. However, SIFT is computationally expensive on datasets and lacks robustness to rotations, scale changes, etc. Literature [7] proposed ThinCrack U-Net, a novel variant of convolutional neural network, which improved performance on the CrackTree260 dataset by optimizing the loss function and combining U-Net components. Yet, this method lacks in-depth exploration of its generalization ability in other datasets or real road environments. Literature [8] pointed out that DeepLabv3 network has higher computational complexity, limiting its application in resource-constrained environments such as mobile devices or real-time systems. However, Zhuang et al. [9] noted that the success of most deep learning models in semantic segmentation comes at the cost of heavy computational burden.

YOLO-based methods combine Backbone, Neck, and Head to regress bounding boxes and classify each crack category [10]. Mandal et al. [11] applied YOLO series networks to crack detection, achieving good results on the test dataset of the IEEE Global Road Damage Detection Challenge. Despite the contributions of the above studies to road damage detection tasks, they share a common issue. The competition does not require detection speed, only accuracy as an evaluation criterion, resulting in models with large parameter sizes and high computational costs. Therefore, these algorithms are not suitable for lightweight edge computing devices. Reference [12] proposed a novel Lightweight Adaptive Dynamic Focus Convolutional Neural Network (LAND-FCNN), optimizing backbone networks through partial convolution and batch interactive attention to improve inference efficiency and address limited sample data issues. PCTNet [13] optimized pixel-level crack segmentation through hierarchical structures of cross-scale patch embedding layers and dual attention transformation blocks, reducing computational costs and improving accuracy. Zhang et al. [14] proposed a lightweight artifact pose measurement algorithm based on the YOLO framework, achieving pose measurement through lightweight backbone networks, rotating anchors, and two-stage fine-tuning strategy.

The studies mentioned above provide references for lightweight road damage detection models, but there is still room for further optimization in terms of model lightweighting and detection accuracy. This paper proposed a lightweight and fast detection method based on YOLOv8 (YOLOv8-LF). This method is more lightweight, capable of fully utilizing semantic information, while improving detection accuracy. The specific innovations are as follows.

1. In this paper, the CG block module was introduced into the Backbone section of YOLOv8 to capture local features, surrounding context, and global context, and integrate these pieces of information. This module enhanced the model's perceptual ability for input data, constructing a new backbone feature extraction network.
2. To reduce the computational complexity of the model, this paper introduced the mixed convolution GSConv into the Neck section of YOLOv8. This not only lowered the computational load but also further enhanced accuracy.
3. Addressing the uniqueness of crack shapes and aiming to fully integrate information from different stages, this paper further introduced the cross-stage local network VoV-GSCSP into the Neck section of YOLOv8.

The structure of this paper is as follows. The first section introduces the current research status on crack detection, covering mainstream methods, technological challenges, and briefly outlines the innovations of the proposed model. The second section reviews relevant literature and previous work, particularly focusing on recent research relevant to the approach in this paper. The third section provides a detailed description of the overall network architecture of the proposed method and analyzes its theoretical advancements. The fourth section analyzes the experimental results and comparative studies conducted on the RDD-2022 dataset. The fifth section discusses the advantages and limitations of the proposed model. The sixth section summarizes the research outcomes and discusses future development trends.

## 2 Related work

### 2.1 Traditional detection methods

Traditional crack detection methods include threshold-based methods [15] and edge-based methods [16]. Threshold-based methods typically distinguish crack regions from non-crack regions by setting a threshold for gray values or other feature values. However, these methods are prone to failure under varying lighting conditions and exhibit poor robustness. Edge-based methods identify cracks by detecting edges in the image. These methods work well when the crack edges are distinct but perform poorly for small or blurred cracks. Lu et al. used pulse air flow thermography to detect and evaluate cracks on sample surfaces [17]. In another study, Ai et al. [18] achieved precise crack detection by combining probabilistic graphical calculations and multi-scale neighborhoods of crack pixels using a probabilistic graphical model (PGM) and support vector machine (SVM). This method has a long computation time when processing large-scale images, making it difficult to meet the requirements for real-time detection. Cho et al. [19] detected cracks in concrete structures using methods such as width transformation, aspect ratio filtering, and crack region search. Although this method performs well in practical applications, its ability to recognize complex crack shapes is limited. Othman et al. [20] achieved crack detection using an improved Otsu-Canny edge detection algorithm. However, the improved algorithm still has limitations in handling high-noise images and requires further improvements to enhance its noise resistance. Although these traditional image processing methods can effectively detect cracks, the crack features need to be manually designed, and the computational complexity results in poor real-time performance, making it difficult to meet the requirements of actual pavement maintenance.

### 2.2 Deep learning methods

To overcome the problem of manual feature extraction in traditional methods not adequately representing cracks, deep learning methods can automatically extract various features of cracks. Reference [21] proposed a Region Proposal Network (RPN) that generates high-quality region proposals almost cost-free by sharing full-image convolutional features with the detection network, significantly improving the speed and accuracy of crack detection when combined with Fast R–CNN. Pham et al. [22] proposed a method combining deep learning and image processing techniques to achieve automatic identification and size measurement of ground cracks, improving both accuracy and processing speed. Liu et al. [23] conducted integrated learning of YOLOv4 and Faster R–CNN, using semantic segmentation as an enhancement method to construct a road interest map. Wang et al. [24] proposed an end-to-end pavement crack detection network based on Swin-Transformer, more accurately describing pavement cracks by modeling long-distance interactions and adaptive spatial aggregation. Reference [25] proposed a novel unsupervised generative adversarial network that can generalize well to tunnel images with complex lighting, addressing the problem of low-light enhancement in tunnel surface defect detection. Su et al. [26] proposed MOD-YOLO, successfully solving the problems of channel information loss and insufficient receptive field. Reference [27] introduced the latest Transformer module [28] into YOLOv5, effectively improving the accuracy of crack detection. Diao et al. [29] introduced the global shuffle attention module and non-parametric attention feature fusion module (PAFF) into YOLOv5, which not only improved computational speed but also significantly reduced the model parameter size. Xiang et al. [30].

proposed a segmentation method combining pyramid structure and dilated convolution to enhance feature extraction capability. Ma et al. [31] proposed a lightweight network based on the YOLO v5 architecture, YOLO v5-DE, which employs efficient convolutions and dense feature connections to achieve narrow crack detection with low computational complexity. However, this method is only applicable to cracks captured at close range.

YOLOv8 is currently the most advanced YOLO model, but it still has some shortcomings in crack detection. First, YOLOv8 tends to exhibit missed or false detections. This is mainly because it divides the input image into smaller grids, with each grid only responsible for predicting one object. This approach fails to fully utilize contextual information. Second, the YOLOv8 model [32] is relatively large, requiring high computational resources and substantial storage space. The Neck component of YOLOv8, which connects the Backbone and Head networks, is responsible for feature fusion and processing. In traditional convolutional neural networks, the processes of spatial compression and channel expansion often result in the loss of some semantic information [33]. The literature [34] has improved the YOLOv8 model by enhancing its loss function and backbone network to achieve small object detection. Wang et al. [35] restructured the Neck of YOLOv8s by incorporating the BiFPN concept, achieving efficient optimization of the model. We have also introduced various testing techniques to improve crack detection performance.

## 3 YOLOV8-LF method

Our method focused on improving the backbone and neck networks of YOLOv8 to create a lightweight, semantically enhanced detection model. The overall architecture of YOLOv8-LF is shown in Fig. 1. The network primarily consisted of three components, namely, Backbone, Neck, and Head. In the Backbone, this paper integrated the Context Guided Block (CG block) module for feature extraction of crack objects; in the Neck, two new modules were introduced to enhance the performance of fused localization and classification information; in the Head, three detection heads were employed to predict various types of cracks. The numbers on the modules represented the channel numbers of the input feature maps.

**Fig. 1:** Overall structure of the YOLOv8-LF method.

### 3.1 The backbone network

To comprehensively consider the context and improve the accuracy of model detection, this paper introduced the CG block into the backbone network of YOLOv8. The CG block [36] includes four key feature extractors, as shown in Fig. 2(a): the local feature extractor Floc, the surrounding context extractor Fsur, the joint feature extractor Fjoi, and the global context extractor Fglo.

**Fig. 2:** Schematic diagram of CG Block feature extractors.

Firstly, Floc and Fsur were used to learn local features and their corresponding surrounding context. Floc is a 3 × 3 standard convolution layer that learns local features from adjacent feature vectors. Fsur is a 3 × 3 dilated convolution layer, as dilated convolution has a larger receptive field and can efficiently learn surrounding context. Therefore, the joint feature is represented by Formula 1:

(1) $$F_{joi}\left(f\right)=P\text{Re}LU\left(BN\left(F_{loc}\left(f\right)\|F_{sur}\left(f\right)\right)\right)$$

In the equation, || denotes the concatenation operation, BN represents batch normalization, and PReLU denotes parametric ReLU.

In the second step, *Fglo* was utilized to extract global context to enhance the joint feature. *Fglo* consists of a global average pooling layer for aggregating global context, and subsequently these global context information was further extracted by a multilayer perceptron. The calculation formula for global context is:

(2) g=δ(MLP(GAP(f)))

In the equation, δ denotes the sigmoid function, and GAP represents global average pooling.

Finally, using a scaling layer, the re-weighted joint feature was obtained by reweighting the extracted global context. The operation of Fglo is adaptive to the input image, as the global context is extracted from the input image. The formula for calculating the re-weighted joint feature is given by Equation (3):

(3) $$F^{\prime }=F⊗g$$

Where ⊗ denotes element-wise multiplication.

Fig. 2(b) illustrates that the CG block module can capture contextual features at all stages, fully leveraging information from both semantic and spatial hierarchies. The semantic information was fully used by the model, which was crucial for accurately classifying each pixel in.

the image. This paper improved the YOLOv8 with the proposed CG block to obtain a better backbone feature extraction network. The new backbone network simultaneously captured local features, surrounding context, and global context and then integrated the information to improve the accuracy of semantic segmentation, which improved the feature capture and learning capabilities of the backbone network.

### 3.2 The neck network

Li et al. [37] proposed the GSConv module, which combines depth-wise separable convolution with the channel shuffle operation from ShufeNet [38]. The structure of the GSConv module is illustrated in Fig. 3. The feature branch adopted a design philosophy of increasing and then reducing dimensionality, ultimately achieving information exchange between features through concatenation and channel reordering. Compared to the backbone network, the feature maps outputted by the backbone in the neck network have smaller dimensions but more channels, which facilitated smoother feature transformation and propagation, effectively preserving semantic information. Therefore, YOLOv8-LF incorporated the GSConv module into the neck network to reduce computational complexity.

**Fig. 3:** Structural diagram of the GSConv module.

The feature map received by the GSConv module first underwent a standard convolution with a stride of 1 and a kernel size of 1, adjusting the channel number to half of the output channel number. Subsequently, the resulting feature map was fed into a depth-wise separable convolution (DWConv) with a kernel size of 5 and a stride of 1 [37]. Next, the output feature map of DWConv was concatenated with the output of the standard convolution. Finally, a channel shuffle operation was applied to the feature map obtained in the previous step to generate the final output feature map. GSConv combines standard convolution and depthwise separable convolution, retaining sufficient feature information while significantly reducing computational complexity. This design allows the YOLOv8-LF model to handle complex tasks more lightweight and efficiently.

In addition, Li et al. [37] used the one-shot aggregation method to design the cross stage partial network (GSCSP) module, VoV-GSCSP. The module combined the Coordinate Attention (CA) module with GSConv technology. The Coordinate Attention module initially decomposed channel attention into two one-dimensional feature encodings along the width and height of the feature map, then aggregating information by summarizing features in each spatial direction. This structure effectively guided attention, enhancing the network's sensitivity and localization capability towards targets. Fig. 4 illustrates the partial network of the VoV-GSCSP module.

**Fig. 4:** The schematic structure of the VoV-GSCSP module.

The VoV-GSCSP module, through the Coordinate Attention module, promotes the effective fusion of information from multiple feature maps in both spatial and channel dimensions. This efficient transmission and interaction of information enable the network to more accurately localize targets. Additionally, the introduction of the Coordinate Attention module enhances the network's perception capability towards targets without adding extra computational burden. The application of this structure in the neck network of YOLOv8-LF effectively balances the relationship between computational complexity and network performance.

### 3.3 The detection head

The feature map generated by the Neck network of YOLOv8-LF was fed into the detection head [32] for prediction. This section included three detection heads, with each detection head responsible for detecting objects of different scales and sizes. The structure of the detection head is illustrated in Fig. 5.

**Fig. 5:** Schematic diagram of the detection head structure.

The detection head separated the regression branch from the classification branch. The regression loss computation consisted of two parts: Clou Loss (CIOU) and Distribution Focal Loss (DFL). Specifically, CIOU Loss was used to calculate the IoU between the predicted box and the target box. Considering that the true distribution usually does not deviate too far from the annotated position, DFL was selected to optimize the probabilities near the label *y* and the two adjacent positions (*y*_*i*_ and *y*_*i+1*_), so that the network distribution focused on the vicinity of the label value, as shown in Equation (4):

(4) $$DFL\left(S_{i,}S_{i+1}\right)=-\left(\left(y_{i+1}-y\right)\log\left(S_{i}\right)+\left(y-y_{i}\right)\log\left(S_{i+1}\right)\right)\text{.}$$

*S*_*i*_ represents the probabilities of the left and right positions, *y*_*i*_ and *y*_*i+1*_, near the label value *y* in the probability distribution outputted by the network.

DFL and CIOU loss were used in combination. DFL was used to calculate the loss of the box distribution probabilities and the distribution probabilities of the labels, optimizing each edge accordingly. The box distribution probabilities were then restored to predicted boxes, and the CIOU loss was used to calculate the loss between the predicted boxes and the actual boxes of the labels, optimizing the predicted boxes as a whole.

Binary Cross-Entropy (BCE) was utilized as the classification loss, determining for each category whether it belonged to that class, and outputting confidence scores accordingly. as shown in Equation (5):

(5) $$BCE=-\frac{1}{N}\sum_{i=1}^{N}\left[y_{i}\cdot \log\left({\hat{y}}_{i}\right)+\left(1-y_{i}\right)\cdot \log\left(1-{\hat{y}}_{i}\right)\right]\text{.}$$

In this formula, N represents the number of samples. yi is the actual label, which takes a value of 0 or 1. ${\hat{y}}_{i}$ is the model's predicted value, representing the probability that the sample belongs to the positive class. The detection head directly outputted confidence scores for each class, and then took the maximum value as the confidence of this anchor box.

YOLOv8-LF includes three detection heads, each responsible for detecting cracks at different scales. The multi-scale detection head design allows the network to detect cracks at various resolutions, thereby improving detection accuracy for cracks of different shapes and sizes. Additionally, the detection heads separate the regression branch from the classification branch. The regression branch focuses on accurately predicting the bounding boxes of cracks, while the classification branch focuses on correctly identifying the crack categories. The introduction of the CIOU and DFL loss functions further enhances the accuracy of the bounding box predictions, ensuring that the detection boxes closely fit the actual crack boundaries. The optimization of the classification branch ensures that each detection box can be accurately classified as a crack, improving the overall detection accuracy. These improvements enable YOLOv8-LF to achieve higher precision and robustness in crack detection tasks, making it better suited for complex real-world applications.

## 4 Experiments and results

The experimental environment was Windows 10, and the model algorithm was implemented based on the PyTorch deep learning framework. The GPU used was an NVIDIA RTX A2000 with 8 GB of VRAM, and the CPU was an Intel(R) UHD Graphics 770. The initial input image size was set to 640 × 640, the model was trained for 200 epochs, and the batch size was set to 4. The initial learning rate was set to 0.03, with a cyclic learning rate of 0.15, and the learning rate momentum remained at the default value of 0.938. The weight decay parameter, warm-up epochs, and warm-up momentum were set to their default values of 5 × 10⁻⁴, 3, and 0.75, respectively. Optimization functions included CIOU, DFL, and BCE. During training, a cosine annealing strategy was employed, and data augmentation methods aligned with those used in the original YOLOv8n model. A table containing the environmental parameter and hyperparameter is shown in Table 1.

**Table 1:** The parameters of all modules.

Environmental parameter and hyperparameter	Value
Operating System	Windows 10
Deep Learning Framework	PyTorch
GPU	NVIDIA RTX A2000 (8 GB VRAM)
CPU	Intel(R) UHD Graphics 770
Input Image Size	640 × 640
Training Epochs	200
Batch Size	4
Initial Learning Rate	0.03
Cyclic Learning Rate	0.15
Learning Rate Momentum	0.938 (default)
Weight Decay Parameter	5 × 10⁻⁴ (default)
Warm-up Epochs	3 (default)
Warm-up Momentum	0.75 (default)
Optimization Functions	CIOU, DFL, BCE
Learning Rate Strategy	Cosine Annealing Strategy
Data Augmentation Methods	Align with original YOLOv8n model

### 4.1 Dataset for the experiment

The dataset used in this study was the publicly available road damage dataset RDD-2022 [39]. The images include perspectives from UAVs and handheld vehicle cameras, enhancing the model's generalization capability in real-world scenarios. In addition to road damage, the dataset initially contained various forms and background images unrelated to the experiment, necessitating image and label processing to exclude non-target content. Through analysis and processing, we selected 2400 images that specifically focused on the target of this experiment.

During dataset handling, we partitioned the data in a 9:1 ratio, comprising 2160 images for the training set and 240 images for the validation set. Additionally, 1 % of background images were added to the training set to enhance dataset composition and realism. The test set comprised images from the RDD-2022 challenge dataset as well as images captured by handheld cameras. As shown in Fig. 6, the research primarily focused on five types of damages: transverse crack D10, longitudinal crack D00, grid crack D20, pit groove D40, and road maintenance Repair.

**Fig. 6:** Five types of damages.

### 4.2 Evaluation parameters

When evaluating the algorithm's performance, two main aspects were considered: accuracy and computational cost. Accuracy was assessed using parameters such as precision, recall, F1−score, average precision (AP), and mean average precision (mAP). The specific calculation methods for these evaluation parameters are as follows:

(6) $$precision=\frac{TP}{\left(TP+FP\right)}\text{.}$$

(7) $$recall=\frac{TP}{\left(TP+FN\right)}\text{.}$$

(8) $$F1-score=\frac{2*precision*recall}{precision+recall}\text{.}$$

(9) $$AP=\sum_{k=0}^{k=n-1}\left[recall\left(k\right)-recall\left(k+1\right)\right]*precision\text{.}$$

(10) $$mAP=\frac{1}{n}\sum_{k=1}^{k=n}AP_{k}\text{.}$$

Here, TP represents the number of true positive samples, TN represents the number of true negative samples, FP represents the number of false positive samples and FN represents the number of false negative samples, and *n* is the total number of categories of detected targets.

In terms of computational cost, it is mainly measured by the number of parameters (Params) and operations per second (GFLOPS). Parameters refer to the number of learnable weights in the model, serving as a key indicator of the model's complexity and size. GFLOPS measure the computational complexity of the model, representing the number of floating-point operations required per second, which reflects the model's computational demand. FPS indicates the inference speed of the model, which is crucial for real-time applications, showing how many frames the model can process per second. Smaller values for Params and GFLOPS indicate that the model requires fewer computational costs and hardware resources [40]. Frames per second (FPS) is calculated by measuring the detection response time, as shown in Equation (11):

(11) $$FPS=\frac{1}{Time},Time=Tp+Ti+Tn\text{.}$$

Where Tp represents the image preprocessing time, Ti represents the inference time, and Tn represents the post-processing time.

### 4.3 Experimental results

The precision and recall rates of the model presented in this paper are relatively balanced across various categories, indicating that the detection performance of the model is consistent across all categories without significant bias. Table 2 shows the different detection results for the five categories. Additionally, the method proposed in this paper has significantly improved the accuracy and recall rates in each category, demonstrating that the model has achieved notable enhancements across all categories.

**Table 2:** Different accuracy results of five categories.

class	precision(%)		recall(%)	
	YOLOv8	ours	YOLOv8	ours
D10	60.9	**67.8**	66.3	**72.2**
D00	64.6	**67.6**	58.7	**63.5**
D20	67.6	**87.3**	64.7	**68.6**
D40	62.7	**64.2**	68.2	**75.0**
Repair	60.4	**78.8**	77.2	**80.7**

#### 4.3.1 Backbone network ablation experiment

To comprehensively evaluate the effectiveness of the proposed optimization on the model's backbone network, ablation experiments were conducted to validate the improvements. Firstly, the unaltered YOLOv8 model was taken as the baseline. Subsequently, the modified backbone network, incorporating the CG block module, was introduced as the improved backbone (Case 1). The experimental results are detailed in Table 3.

**Table 3:** Ablation experiment on backbone network optimization.

Models	FPS	GFLOPS	precision(%)	F1-score(%)
YOLOv8	178.5	8.1	77.9	63.2
Case 1	172.4	8.6	**82.2**	**66.6**

The experimental results indicated that after replacing the backbone network, Case 1 achieved a 4.3 % increase in accuracy and a 3.4 % increase in F1 score compared to the unmodified YOLOv8 model. The increase in GFLOPS for Case 1 indicates that the computational performance of the model has improved. Fig. 7 provides a more comprehensive depiction of the accuracy trend of baseline and case 1 when epoch is set to 200, clearly showing the advantage of case 1 over baseline.

**Fig. 7:** Visualization of accuracy results.

In conclusion, this clearly demonstrates the effectiveness of the optimization applied to the model's backbone network in this study. The newly introduced CG block module enables the model to more effectively utilize semantic information, thereby significantly improving detection accuracy. These results provided substantial support for enhancing the model's performance in object detection tasks.

#### 4.3.2 Neck network ablation experiment

In the cervical network ablation experiment, the GSConv module and VoV-GSCSP module were introduced as improvements to the cervical network, resulting in the ablation model (Case2). The detailed experimental results are presented in Fig. 8.

**Fig. 8:** Neck network ablation experiment results.

By observing the experimental results in Fig. 8, it is evident that applying both the GSConv module and the VoV-GSCSP module at the bottleneck of YOLOv8 can significantly reduce the model parameters. This finding emphasizes the successful optimization of the bottleneck network in this study. It is noteworthy that this implies the successful lightweighting of the model while maintaining its performance level. These improvements are not only expected to enhance the practicality of the model but also indicate the positive impact of optimizing the bottleneck network on the overall performance of the model. Fig. 9 presents the detection outcomes for three cases, and notably, the results for case 2 outperform those for YOLOv8 and case 1. This observation unequivocally underscores the efficacy of the implemented enhancements.

**Fig. 9:** Visualization of experimental results in three cases.

In the table, √ indicates the utilized module.

#### 4.3.3 Comparison of different methods

This study systematically conducted stepwise ablation experiments for all modules and algorithmic optimizations. YOLOv8-LF represented the ultimate model integrating all the designed modules and algorithmic optimizations proposed in this paper. Experimental data is presented in Table 4.

**Table 4:** Stepwise ablation experiments.

Models	CG block	GSConv	VoV-GSCSP	GFLOPS	FPS	Precision(%)	F1-score(%)
YOLOv8				8.1	178.5	77.9	63.2
Case 1	✓			8.6	172.4	82.2	66.6
Case 2		✓	**✓**	7.3	158.7	75.4	61.1
Case 3		✓		8.0	178.6	75.7	62.7
Case 4			✓	7.4	250.0	81.4	66.5
Case 5	✓	✓		8.5	277.0	77.6	64.8
Case 6	✓		✓	7.9	166.7	79.0	64.3
YOLOv8-LF	✓	✓	**✓**	7.8	**294.1**	**84.5**	**67.5**

For this part of the ablation experiments, we used YOLOv8 as the baseline model. Cases 1–6 represent the models obtained by optimizing different modules. From Table 4 and it can be seen that Case 1 has the highest GFLOPS, but its accuracy, F1-score, and FPS are all inferior to YOLOv8-LF. YOLOv8-LF was the final model obtained by applying all modules we designed and algorithm optimizations. Compared to YOLOv8, YOLOv8-LF exhibited significant improvements in overall performance. The FPS has increased by 116, which means that the model can process more images in the same amount of time, thereby accelerating the target detection process and enhancing real-time performance. These data indicate that adopting the YOLOv8-LF model significantly improves the accuracy of the model in target detection tasks, thereby more effectively identifying and locating targets. Additionally, YOLOv8-LF ranks the first in both accuracy and F1 score. In conclusion, these data reflect the optimization of YOLOv8-LF in terms of accuracy, speed, and computational efficiency, making it more competitive in practical applications.

### 4.4 Results of complex road detection

In general scenarios, the specific conditions of roads vary widely, making the robustness of the model particularly crucial. To assess the model's performance under diverse conditions, this paper selected three different scenarios and conducted detailed analyses for each comparative experiment. The unmodified model was referred to as baseline, denoted as YOLOv8. Case 1, incorporating the CG block module into the backbone, was named YOLOv8-CG. Case 2, integrating the GSConv and VoV-GSCSP modules into the neck, was designated as YOLOv8-GV.

Fig. 10(a) illustrates the detection results of common cracks. Observation revealed the presence of false positives in the unimproved model, while the optimized YOLOv8-LF demonstrated higher accuracy and reliability under the same conditions. Detecting cracks with unclear textures posed a more challenging task compared to common crack detection.For the unclear-texture cracks depicted in Fig. 10(b), YOLOv8-GS could identify all cracks, but YOLOv8-LF exhibited a more prominent accuracy, indicating that our optimization algorithm has.

**Fig. 10:** Comparison of detection results of four algorithms in three different scenarios.

effectively enhanced the model's ability to capture contextual information. In Fig. 10(c), detection experiments were conducted using images containing grid cracks and potholes of varying sizes. The results show that only YOLOv8-LF can accurately detect all damages, while other detection algorithms exhibit instances of both false negatives and false positives.

Tree branches, due to their similarity to crack features, were considered background noise in crack detection. In Fig. 11(a), only YOLOv8-LF did not produce false positives. Reduced light and decreased visibility in foggy conditions presented challenges for detecting road damage. In foggy conditions, the impact of local traffic white lines on crack-type damage was magnified, posing significant challenges for feature acquisition and learning algorithms. In Fig. 11(b), only YOLOv8-LF successfully detected longitudinal cracks covered by traffic white lines. Additionally, weather conditions should be considered for accurate detection. For instance, strong light can cast shadows of roadside vehicles, potentially interfering with damage detection. Therefore, we conducted detection experiments using images of transverse cracks with shadows. In Fig. 11(c), only YOLOv8-LF detected the transverse crack area. Therefore, YOLOv8-LF demonstrates higher accuracy and reliability in complex environments.

**Fig. 11:** Visualization comparison of the model's detection results under background noise, foggy weather, and lighting changes.

### 4.5 Comparison experiments

In this paper, the proposed method was compared against SSD [40], DETR [40], YOLOv7-tiny [41], EfficientDet [42], and LE-YOLOv5 [29] through experimental evaluation. Faster R–CNN [43] and Cascade R–CNN [44] are classic and widely-used two-stage detection algorithms, known for their high accuracy and relatively fast speed. SSD and DETR are single-stage object detection algorithms that have been widely applied in recent years. SSD is characterized by its fast detection speed and high accuracy, while DETR significantly enhances detection performance by introducing the Transformer architecture. YOLOv7, proposed in 2022, includes a lightweight version called YOLOv7-tiny, which has become one of the most outstanding lightweight detection algorithms due to its.

excellent performance and smaller model size.As shown in Table 5, compared to YOLOv7-tiny and YOLOv8s, YOLOv8-LF reduces the model size by 50.8 % and 73.5 %, respectively. This significant reduction in size makes YOLOv8-LF more applicable in resource-constrained environments. Additionally, YOLOv8-LF achieves 294 FPS, demonstrating its superior performance in real-time detection tasks and significantly enhancing detection efficiency. In terms of comprehensive evaluation metrics, YOLOv8-LF shows significant advantages in GFLOPS and accuracy. Among all the tested algorithms, YOLOv8-LF maintains top detection accuracy while keeping computational complexity low. These results indicate that YOLOv8-LF not only achieves substantial breakthroughs in model lightweighting but also exhibits robust and reliable performance in practical applications, proving its superiority in various complex road environments.

**Table 5:** Multiple algorithms’ comparison.

Models	Params(M)	GFLOPS	FPS	Precision(%)	Recall(%)	F1-score(%)
YOLOv8s [32]	11.2	28.6	186	79.9	53.6	64.2
Faster R–CNN [43]	41.45	94.4	9	57.0	52.2	54.5
Cascade R–CNN [44]	–	–	–	56.9	49.9	53.2
SDD [41]	26.77	60.7	15	61.8	49.7	55.3
DETR [41]	36.74	100.6	36	48.6	38.3	42.7
YOLOv7-tiny [45]	6.02	13.1	111	51.3	52.5	51.8
Efficient det [42]	3.87	5.2	27	47.1	45.5	46.1
LE-YOLOv5 [29]	3.41	7.0	71	63.9	53.2	58.1
YOLOv8-LF(ours)	**2.97**	7.8	**294**	**84.5**	**56.2**	**67.5**

## 5 Discuss

The experimental phase of this study is divided into two main parts: progressive ablation experiments and multi-model comparative experiments. The ablation experiments show that compared to YOLOv8, YOLOv8-LF improved accuracy by 6.6 %, increased the F1 score by 4.3 %, and achieved 294 FPS. In other model comparison experiments, compared to the excellent lightweight models in recent years, YOLOv7-tiny and YOLOv8s, our model demonstrates significant advantages in accuracy based on a lower number of parameters. Compared to models with higher computational complexity, our model offers a significant reduction in size without compromising accuracy. This means that our model achieves improved performance while being more lightweight.

As shown in Fig. 12, despite YOLOv8-LF being the best-performing model among all, it still exhibits missed detections in scenarios where the crack textures are unclear and the background is complex. Therefore, future efforts should focus on enhancing the model's accuracy and generalization capability in situations involving complex backgrounds and unclear target textures.

**Fig. 12:** Visualization of method limitations.

## 6 Conclusion

An analysis based on existing road damage detection methods, this paper proposed a lightweight ground crack rapid detection method based on semantic enhancement within the YOLOv8 framework. The introduction of the Semantic Segmentation Context Guided Block (CG block) module enhanced the feature extraction network of YOLOv8, significantly improving the model's prediction accuracy. The incorporation of GSConv and VoV-GSCSP modules, while enhancing computational speed, drastically reduced the model's parameters. Finally, the proposed method was extensively tested on the public dataset RDD-2022. Experimental results demonstrate that our approach exhibited stable and effective performance in crack detection tasks. In comparison to the model YOLOv8, the model parameters have been reduced by 73.5 %. YOLOv8-LF achieved a 6.6 % accuracy improvement, a 4.3 % increase in F1-score, and an FPS enhancement from 178 to 294. This validated the method's ability to maintain exceptional robustness and reliability while achieving lightweighting, showcasing its broad potential for application. Therefore, our study provides significant reference value for lightweight road damage detection algorithms, offering possibilities for deploying road damage detection algorithms on lighter edge computing devices.

In the future, several directions can be further explored to expand this work. Firstly, enhancing the model's detection accuracy in scenarios with complex backgrounds and unclear textures. Secondly, there is still potential to improve the model's generalization capability by expanding and optimizing the dataset. Improvements in data collection methods can increase the volume of data related to various types of road damage. Additionally, considerations should be given to expanding the applications of object detection, whether from a lightweight perspective or in terms of post-processing of detection results.

## CRediT authorship contribution statement

**Bing Yi:** Project administration, Resources, Supervision. **Qing Long:** Methodology, Software, Validation, Visualization, Writing – original draft, Writing – review & editing. **Haiqiao Liu:** Funding acquisition, Supervision, Writing – review & editing. **Zichao Gong:** Software, Visualization, Writing – review & editing. **Jun Yu:** Supervision, Visualization, Writing – review & editing.

## Declaration of competing interest

The authors declare that they have no known competing financial interests or personal relationships that could have appeared to influence the work reported in this paper.
